# Dynamic Recognition and Analysis of Gait Contour of Dance Movements Based on Generative Adversarial Networks

**DOI:** 10.1155/2022/3276696

**Published:** 2022-06-08

**Authors:** Junlin Ren, Jae-Keun Park

**Affiliations:** Sangmyung University, Seoul 03016, Republic of Korea

## Abstract

With the generation of images, videos, and other data, how to identify the gait of the action in the video has gradually become the focus of research. Aiming at the problems of complex and changeable movements, strong coherence, and serious occlusion in dance video images, this paper proposes a dynamic recognition model of gait contour of dance movements based on GAN (generative adversarial networks). GAN method is used to convert the gait diagrams in any state into a group of gait diagrams in normal state with multiple angles, which are arranged in turn. In order to retain as much original feature information as possible, multiple loss strategy is adopted to optimize the network, increase the distance between classes, and reduce the distance within classes. Experimental results show that the average recognition rates of this model at 50°, 90°, and 120°are 93.24, 98.24, and 97.93, respectively, which shows that the recognition accuracy of dance movement recognition method is high. And this method can effectively improve the dynamic recognition of gait contour of dance movements.

## 1. Introduction

The posture and movement of a person walking is referred to as gait. The majority of today's gait research focuses on human gait movement. Gait is the only noninvasive method that can be employed, unlike fingerprints, face, and iris. Gait recognition, when compared to other long-distance biometric recognition technologies, has the benefits of long-distance recognition, noncontact, difficult concealment, and so on and has a lot of potential and application possibilities. Few universities or institutions have studied dance movements among the many studies on human body movement recognition, mainly because dance is a way of expressing emotions to the public through body movements, and dance movements in this category also include many dance movements with their own characteristics [1]. As a result, dance movement research is still in the stage of dance movement analysis. Most of the time, the gathered dance movements are gesture analyzed and then adapted to animated character performances utilizing animation processing software.

In order to solve the problem that the training gait cannot meet the training requirements of dance action steps, domestic and foreign scholars have successively carried out research on the generation method of personalized training gait. Qin et al. established the motion trajectory generation models of hip, knee, and ankle joints with multilayer perceptron, respectively [2]; Rida et al. established an ellipse model, which divided the human body into seven parts according to the proportional relation of the center of mass of the ellipse, and modeled each part [3]. Deng et al. proposed the method of deep gait and used the pretraining model VGG-16 to obtain the feature representation of gait map [4]. Li et al. proposed to learn the similarity between gait diagrams directly through the depth CNN (convolutional neural network) and extract the features of gait diagrams through CNN for matching recognition [5]. Zhao et al. extracted the information of human motion shape by Canny edge detection to represent the information of motion edge and then achieved the purpose of human motion recognition by matching similar edges [6]. Hnatiuc et al. changed the traditional separate training and combined attitude estimation and action recognition in order and put forward a framework for combining attitude estimation and action recognition [7]. Luo et al. reconstruct the 3D structure of human beings to generate views and 3D models that can be generated in any 2D by projection, but they usually need to fully control and cooperate in multiple camera environments [8]. However, there are still some shortcomings in the personalized gait generation experiment in the above research: the research object is limited to single or local joints, lacking comprehensive consideration of joint coupling relationship and overall coordination of motion. It is difficult to accurately describe the walking characteristics of human body only by the difference of gait parameters.

The input for recognizing human dance movements must be a series of motions, yet dance movements are similar to other sorts of movements. The activities in the video contain a lot of redundant information, and while the directions of the actions may alter, they can all be considered the same action based on the sequence of events. Traditional dynamic recognition methods based on the approach have a low identification rate, are unable to distinguish joint changes in precise dance motions, and have a poor recognition effect. In light of this shortcoming, this research investigates a GAN-based dynamic recognition and analysis method for dance movement gait contour (generative adversarial networks). The global coordination of the generated gait and whether it fits the standards of naturalness, adaptability, and stability are investigated using the gait stability criterion, which is based on the notion of human balanced perception. We intend to develop a tailored gait generation approach that can accurately represent distinct human gait features and give theoretical support for personalized training as a result of this research.

### 1.1. Innovation of This Paper

1. In order to extract effective gait features for cross-view gait recognition, this paper proposes a cross-view gait feature extraction method based on GAN, which only needs to train a model to transform the gait template into any view. Retain the original identity information to the greatest extent, thus improving the accuracy of gait recognition.
2. In this paper, GAN is used to transform the gait map, and a GAN recognition model is proposed to make full use of the feature information of the gait map, thus improving the accuracy of gait recognition.

### 1.2. Organizational Structure of This Article

The first chapter introduces the research background and significance, and then introduces the main work of this paper. The second chapter mainly introduces the related technologies of gait contour dynamic recognition of dance movements. The third chapter puts forward the specific methods and implementation of this research. The fourth chapter verifies the superiority and feasibility of this research model. The fifth chapter is the summary and prospect of the full text.

## 2. Related Work

### 2.1. Overview of GAN Research

With the innovation of information technology and the constant replacement of computing power of hardware devices, artificial intelligence [9–11] is developing vigorously in the information society, and the field of machine learning represented by generative model continues to attract researchers' attention.

The performance of GAN model proposed by Vma and others in generating image data surprised researchers. At present, its research in computer vision, medicine, natural language processing, and other fields has been active. It shows that there are few summary papers on the structure and performance of GAN at present, and other research work mainly focuses on the performance verification of different types of GAN architectures. Because the benchmark data set cannot reflect the diversity well, the comprehensive discussion of GAN in these works is limited. Paulo et al. proposed a GAN framework based on FC layer modeling, which only showed high performance in a few groups of data distribution. The deep convolution GAN model proposed by Switonski et al. can smooth the training process of generator and discriminator and contribute to improving the stability. Creswell et al. proposed a framework based on GAN, called Fu-sionGAN, which generates a fused image by controlling two input images [12]. Experiments show that the fusion method can change the shape and features of the input image and generate a new image while retaining the main content of the input image. Wang et al. summarized the image super-resolution technology based on deep learning and divided it into three types: supervised, unsupervised and specific application fields, and provided systematic super-resolution theory and practical methods [13]. Lei et al. proposed a framework that can be used to decipher passwords, so that GAN can be applied to decipher passwords [14]. In addition to the above areas, GAN has been successfully applied in other directions, such as domain adaptation, sequence generation, semi-supervised learning, semantic segmentation, attack resistance, machine translation, automatic driving, and so on.

### 2.2. Research Status of Gait Recognition

In recent years, gait recognition has attracted more and more attention in video surveillance and computer vision fields such as crime prevention and forensic identification, and its development will greatly promote the development of application, society, and computer vision. Therefore, gait recognition will become more and more important in the future. Unfortunately, gait recognition is still a challenging task because it has many potential sources of change, such as angle change, transportation, and clothes change.

Mosser et al. put forward the application of single linear projection, called view invariant discriminant projection, whose single property enables cross-view gait recognition without knowing the query gait view [15]. Lu et al. used the stacked progressive automatic encoder to convert the angle and converted the arbitrary angle of gait features into a single side view angle [16]. Yao et al. used 2D stick map obtained by connecting nine body points extracted from gait to simulate human movement [17]. Cai and others simulated human legs and used them to analyze human walking and running [18]. The research of Gadaleta et al. also simulates human legs, in which the legs are represented by many thick lines connected at one point [19]. Connie et al. put forward a method to predict 3D pose from 2D pose matching database, which predicts 3D pose according to the mutual constraint relationship of every joint in human body [20].

Gait is periodic, coordinated, and balanced, and the analysis in one cycle of gait can reduce the calculation amount of gait recognition and improve the operation efficiency. Gait periodicity can be analyzed according to the changes of the features of the graphic areas in each frame of binary images, such as area, centroid, and external rectangle. Risi et al. analyzed the periodicity of gait sequence according to the width signal of the binding frame of human body area and proposed a cycle calculation method under the condition of large lateral angle and lateral angle deviation [21]. Zhao et al. used PSO (particle swarm optimization) algorithm to optimize the pattern recognition method of SVM (support vector machine) [22], and the experimental results showed that the recognition rate of PSO-SVM classifier was higher than that of nonparameter optimized SVM classifier for lower limb analysis of five normal walking gait. Mannini et al. used k-nearest neighbor method to classify and recognize gait [23]. DTW (dynamic time warping) is to regularize the motion feature templates with different time lengths according to a certain time warping curve, so as to make the feature templates have the same length and then match them. This method has the advantage of solving the similarity measurement and matching problems of dynamic patterns.

## 3. Methodology

### 3.1. Gait Image Preprocessing

Gait recognition mainly analyzes and processes moving image sequences containing people, which usually includes four stages: target segmentation, feature extraction, feature processing, recognition, and classification. It should be noted that gait itself and compared with other biometric technologies also have many shortcomings, which are mainly influenced by emotion, object use, and gait angle. At present, most gait recognition algorithms use cameras to acquire gait data and use two-dimensional methods for gait recognition. In order to improve the recognition effect, the application of multicamera gait recognition algorithm and 3D method can be studied. By using multiple cameras, the problem of feature extraction caused by occlusion can be improved, and 3D modeling of human motion can extract the gait features [18] of human body more accurately and realize more complex feature matching. Multicameras and 3D methods are also the trend of human body recognition. If a motion sequence does not have a separate background picture, we must get the backdrop of motion sequence images [20] in order to collect some local photographs as background images in preparation. It should be noted that the light intensity has a significant impact on the background map selection, and the data of the background map vary substantially depending on the light intensity. Multiple backdrop photos should be picked and collected for optional use to eliminate this influence.

The volume contour area also appears in its own contour area, so there will be repetition in the calculation. Because of the noise in these small areas, the edge tracking algorithm cannot work smoothly, so we must use image connectivity algorithm to remove these small areas and get pure object images. There are many marked points to be extracted in the image sequence and other background noises. In order to extract the target points from multivalued digital images, binarization must be performed.

That is, by setting a threshold *T* [11], the image data are divided into pixel groups larger than *T* and pixel groups smaller than *T* with different values, respectively, so as to extract the feature points we care about, as shown in formula 1:

(1) $$\begin{array}{c} I_{B}\left(u,v\right)=\left\{\begin{array}{c} 255,\begin{array}{cc} \; & I_{P}\left(u,v\right)>T, \end{array}\\ 0,\begin{array}{cc} \; & I_{P}\left(u,v\right)<T, \end{array} \end{array}\right. \end{array}$$

where *I*(*u*, *v*) represents the pixel value of a certain point in the image.

After binarization, the image sequence has only two areas: bright and dark, in which the marked points are bright. By programming and calling the function library, we can get the coordinates (*u*, *v*) of the center of each marked point in the forward process. In the sagittal plane of human body, the distance between waist and hip joint is measured as *D*_*mm*_, and the number of pixels between these two points is obtained as *d* in the image plane, and the corresponding proportional relationship between the two coordinate planes is obtained as follows:

(2) $$\begin{array}{c} s=\frac{D}{d}. \end{array}$$

Therefore, the coordinates of the image plane are converted to the coordinates *x*, *y* of the sagittal plane of the human body, and the change curve of the displacement of the subject's arch in *x*, *y* direction is obtained, as shown in Figure 1:

In this paper, the gait energy map is used as the gait template [16], and the gait energy map can be obtained by averaging the gait contour maps in the gait sequence, which can effectively retain the feature information during walking. As shown in Figure 2, the brightest pixel in the gait energy map represents the highest frequency of the position in the whole gait sequence.

The degree of coordination of human joint movement directly affects the stability of gait when walking, so the author's previous results are used to analyze the stability of the generated gait [18], thus reflecting its overall coordination. With the passage of time, the coordinates of the soles of the feet in two directions are extracted, and then the trajectory of the soles of the feet in two directions is fitted by the least square curve fitting method. The trajectory described by polynomial is to calculate the first derivative to get the gait speed curve of normal walking.

### 3.2. Dynamic Recognition of Gait Contour of Dance

#### 3.2.1. Gait Feature Extraction Based on GAN

Human posture characteristics are derived from human posture information, which can be obtained in two methods. The first is to use attitude estimation on the test set to retrieve the position of human joints and calculate the joint angle; the second is to utilize the coordinates of each joint of the human body received when the motion capture equipment gathers the dance video. Most dance moves involve two arms and two legs, although there is no definite correlation between arms, arms and legs, and legs. The full-body region was chosen because various activities, such as those performed by the actor from bottom to top as a whole, turning about, strolling around, and so on, should be judged and identified by the motion information of the actor's entire body. By partitioning the human body area by the human body position, the impact of garment occlusion on motion recognition can be decreased. The background information with little or no change in the image can also be filtered according to the optical flow value in the process of optical flow feature extraction, so the areas where the information is finally retrieved are the upper body, lower body, and the entire actor's body. As a result, some features of the source gait map may not be effectively reflected in the gait map generated after the conversion due to angle conversion. As the angle difference grows, more feature information in the source gait map is masked, and the amount of feature information in the source gait map that can be expressed by the converted gait map decreases, resulting in a lower recognition rate.

In the experiment, the camera is stationary, and people walk in front of the camera without being blocked by objects. Therefore, contour extraction is essentially to eliminate the background from the sequence images to obtain the contour of the moving target. Its implementation steps are as follows:

1. Because the scene is approximately still in the whole video sequence, the background corresponds to low-frequency information. Therefore, the average value of pixels in sequential images can be used to estimate the static background.
2. Background difference method is used to detect moving targets in sequence images, and binary segmentation of images is performed under a set threshold.
3. The contour information of the moving person in the sequence image is further extracted by the inner boundary tracking algorithm.

In order to eliminate the inconvenience of feature extraction caused by motion change, the centroid points of human body contour are calculated, respectively, and used as the coordinate origin of the image.

Let (*x*_*c*_, *y*_*c*_) be the centroid coordinate, *N*_*b*_ be the total number of boundary pixels, and (*x*_*i*_, *y*_*i*_) be the pixels on the boundary, then

(3) $$\begin{array}{c} \left\{\begin{array}{c} x_{c}=\frac{1}{N_{b}}\sum_{i=1}^{N_{b}}x_{i},\\ y_{c}=\frac{1}{N_{b}}\sum_{i=1}^{N_{b}}y_{i}. \end{array}\right. \end{array}$$

In order to eliminate the influence of image scale and signal length on the training and recognition process, the minimum-maximum normalization method and equally spaced resampling method are used to reduce the amplitude and length of the signal, respectively. The prediction of 3D pose mainly depends on the identification and planning of each person's crossing angle. It is difficult for us to predict 3D posture, which requires a lot of work and research. The 2D pose is drawn on the image plane. When the view changes, the 2D pose will change greatly, so it will not resist the change of viewpoint. The solution proposed in this paper is to estimate 3D pose from 2D pose.

After getting the 3D pose, we still need to do normalization, and there are 14 3D joint points. The length unit is the distance from the neck to the center of the hip, the position of the hip is in the center of the left and right hips, and the neck is at the origin of the plane coordinate system. So the joints of the body are normalized as follows:

(4) $$\begin{array}{c} J_{i}^{\prime }=\frac{J_{i}-J_{\text{neck}}}{H_{nh}}, \end{array}$$

_where_*J*_*i*_ ∈ *R*^2^ is the position *i* of body joints, *J*_*i*_′ is the position of *J*_*i*_ after normalization, *J*_neck_ is the position of neck, and *H*_*nh*_ is the distance between neck and hip.

The postures from three different individuals after normalization are shown in Figure 3, from which we can find the differences of leg movement patterns among three different individuals.

Figure 4 shows the flow chart of the whole algorithm.

First, all the gait video sequences of test set, training set, and verification set are uniformly processed into the same gait template. Then, *z*^*p*^ is converted from perspective *a* to perspective *b* through a perspective converter *V* and the feature implicit representation *z*^*g*^=*V*(*z*^*p*^, *a*, *b*) after perspective conversion is obtained.

Finally, it is determined that the identity of *p*^*a*^ is in the verification set of perspective *b*, and the calculation formula of nearest neighbor classifier is as follows:

(5) $$\begin{array}{c} x=\arg\min{\left\|{\hat{z}}^{g}-z_{i}^{g}\right\|}_{2},i\in \left\{1,2,\cdots ,n\right\}. \end{array}$$

Here, ‖·‖_2_ stands for *L*_2_ norm.

#### 3.2.2. Motion Gait Contour Tracking

An important clue to determine the intrinsic movement of pedestrians is the change of human body contour with time. In order to eliminate the information redundancy and reduce the computational complexity, we convert the two-dimensional contour shape changes into one-dimensional distance signals to approximate the spatiotemporal change pattern of gait movement.

The target movements of the dance gait contour extracted during the dance process are divided into heel strike stage, load-bearing reaction stage, middle support stage, end support stage, start stage, prestart stage, swing stage, initial swing stage, middle swing stage, and finally swing stage, when the heel touches the ground again and waits for 9 time periods [7]. In the actual dance process, these nine time periods will appear repeatedly with each point in Figure 5, showing certain regularity and periodicity.

Taking the top edge point as the reference starting point, the contour boundary is expanded counterclockwise to become a one-dimensional signal composed of the distance from the boundary pixel point to the centroid.

(6) $$\begin{array}{c} d_{i}=\sqrt{{\left(x_{i}-x_{c}\right)}^{2}+{\left(y_{i}-y_{c}\right)}^{2}}. \end{array}$$

In order to eliminate the influence of image size and signal duration on the training and recognition process, we normalize the signal amplitude and duration, respectively. When normalizing the amplitude, we divide each distance signal by the maximum value of the distance, so that its value is between 0 and 1. For length normalization, we use equally spaced sampling to make the number of edge points within a certain range, such as 400.

#### 3.2.3. Dynamic Contour Recognition

The input of the authenticity discriminator network is an image, which can come from the sample generated in the target domain or the image in the source domain. The goal of this discriminant model is to learn a classifier to separate the two types of samples as much as possible. Through the contradiction training between the generated model and the generated model, the generated model can generate samples with source domain attributes as much as possible.

That is, the authenticity discriminator acts on the generation network to generate realistic images, where *I*^*i*^ is the source image and ${\hat{I}}^{i}$ is the sample image generated by the generator. Here, the discriminator generates a probability to indicate whether the image is true or not, and its loss function *L*_*D*_^*R*^ is expressed in the form of cross entropy as follows:

(7) $$\begin{array}{c} L_{D}^{R}\left(I\right)=-t\cdot \log\left[D_{R}\left(I\right)\right]+\left(t-1\right)\cdot \log\left[1-D_{R}\left(I\right)\right],\\ s\cdot t\cdot \begin{array}{cc} \; & t=\left\{\begin{array}{c} 1\begin{array}{cc} \; & \text{if }I\in \left\{I^{i}\right\}, \end{array}\\ 0\begin{array}{cc} \; & \text{if }I\in \left\{{\hat{I}}^{i}\right\}. \end{array} \end{array}\right. \end{array} \end{array}$$

Because of the uncertainty of the target, an extra loss function is needed at the top of the generator to restrict the generated target image, and an independent network named domain discriminator is connected at the top of the converter. The discriminator takes the source image and the target image as inputs and is trained to generate the scalar probability of input-to-correlation.

Gait is a space-time movement, so we expect to use STC (spatiotemporal correlation) to capture its spatial structure characteristics and time translation characteristics.

For any two gait sequences, after the above processing, they are converted into distance signal sequences *I*_1_(*t*), *I*_2_(*t*); The feature space [*ℓ*_1_, ⋯, *ℓ*_*k*_] is constructed, and their projection trajectories *P*_1_(*t*), *P*_2_(*t*) in the feature space are as follows:

(8) $$\begin{array}{c} P_{1}\left(t\right)={\left[\ell_{1},\cdots ,\ell_{k}\right]}^{T}I_{1}\left(t\right),\\ P_{2}\left(t\right)={\left[\ell_{1},\cdots ,\ell_{k}\right]}^{T}I_{2}\left(t\right). \end{array}$$

Then the similarity measure between them can be defined as

(9) $$\begin{array}{c} d^{2}-\underset{ab}{\min}{\sum_{i=1}^{T}\left\|P_{1}\left(t\right)-P_{2}^{\prime }\left(at+b\right)\right\|}^{2}. \end{array}$$

Among them, *P*_2_′(*at*+*b*) is the vector trajectory that is dynamically normalized according to time expansion and shift, and the selection of parameter *a*, *b* depends on the change of velocity and phase between different sequences, respectively.

For the training of generators and discriminators, we adopt the common confrontation loss, and the formula is as follows:

(10) $$\begin{array}{c} \min_{G}\max_{D}L_{\text{adv}}=E\left[\log D\left({\hat{y}}^{b}\right)\right]+E\left[\log\left(1-D\left(G\left(V\left(E\left(p^{a}\right)a,b\right)c\right)\right)\right)\right]. \end{array}$$

Among them, *E*, *V*, *G*, *D* represents encoder, angle converter, generator, and discriminator, respectively, *p*^*a*^ is the original input gait energy map from *a* angle of view, *c* represents the unique thermal coding of walking state, and ${\hat{y}}^{b}$ is the real gait energy map.

Universal templates representing various categories can be used as template patterns to directly match with test actions for identification. Assume that *x*, *y* represents a certain frame of the test sample and the general template, respectively, which supports the similarity calculation *s*(*x*, *y*):

(11) $$\begin{array}{c} h_{p}^{\prime }\left(x,y\right)=\left\{\begin{array}{c} 1\begin{array}{cc} \; & \text{if }x_{p}\in y_{p}, \end{array}\\ 0\begin{array}{cc} \; & \text{otherwise}. \end{array} \end{array}\right. \end{array}$$

In its calculation process, if the *x*, *y* of the two frames does not match, then *s*(*x*, *y*) is no longer assigned to zero, but a negative value, *h*(*x*, *y*) − 5, is given as a punishment, thus enhancing the differentiation between different actions.

In the process of recognition, each frame of input action should be divided into five parts in turn, and each part should be mapped to the trained cluster. If the key frame is the key frame, we will search the results of each part in its corresponding key table in turn. The real-time action recognition process is shown in Figure 6.

The accumulated scores of these results can be used as the basis for identification, and the end point of the input action pattern and whether it is a legal action can also be judged by matching.

## 4. Experiment and Results

### 4.1. Experimental Data Set and Its Settings

In order to better verify the accuracy of the dance action recognition method designed in this paper, the most commonly used PASCAL VOC 2011-val (Data_P) and Stanford 40 actions (Data_S) data sets [14, 15] and the dance image to be executed (Data_D) are used. After the data collection is completed, use ipi Mocap Studio software to preprocess and correct each frame of the captured contour data. It is defined that the right heel leaves the ground as the gait cycle and the right heel touches the ground as the gait cycle. The gait contour data of 70 dancers were collected.

The generator in this model is an end-to-end unified network, which can be divided into two parts, an encoder and a decoder. The encoder part consists of four convolution layers, which extract features from the source image into a new spatial expression *z*. The extracted features *z* are sent to the decoder, so as to construct the correlation generation target through four decoding layers. We use the generated gait energy map as gait feature. In the testing stage, we trained many models to generate gait energy maps for the test data set and used the nearest neighbor algorithm to calculate the feature recognition rate. The detailed information of encoder and decoder structure is shown in Table 1 and Table 2. The discriminator structure uses four convolution layers.

### 4.2. Experimental Result

After the experiment on the Data_P data set, we selected three methods (ref [17], ref [19], ref [20]) to achieve better recognition results without cross-viewing and compared the average rank-1 accuracy on the same data set. The average rank-1 accuracy in three walking states and all cases is shown in Figure 7.

From Figure 7, it can be seen that the method proposed in this paper has no great advantages over the other three methods in the “running” and “walking” state, but the recognition accuracy is improved in the “jumping” state, which proves that the method proposed in this paper has better adaptability to the interference factor of clothing. In order to verify that actions are divided according to human body structure and consider their advantages, respectively, we have also implemented a case of treating human body actions as a whole in Data_S and Data_D data sets. When the action data are treated as a whole, we choose *θ*=45 as the quantization error of K-means clustering, and the two action data sets after clustering generate an average of 210 and 150 clusters, respectively, in three groups of experiments.  Table 3 compares the recognition results of this method and the method based on whole-body segmentation under two whole-body segmentation schemes.

It can be seen that the classification performance of our method on these two data sets is better than the general body-based pattern, especially on the Data_D data set. This is because the Data_D data set covers basic daily actions, such as running and jumping, which may lead to more changes in the class. Therefore, when these actions are calculated and recognized as a whole, the recognition accuracy will be seriously affected, and our limb-based segmentation method can avoid this shortcoming.

In order to further prove the effectiveness of our method, we also compare it with other commonly used motion recognition methods (DTW, SVM, and PSO). The recognition results of the above methods on the data set are shown in Figure 8.

On the Data_ S data set, the result demonstrates that DTW has the highest recognition accuracy. On these three data sets, the classification performance of SVM and PSO is not as good as this technique. PSO-accuracy SVM's on these three data sets is extremely near to the best score, demonstrating the method's stability and efficacy once again.  Figure 9 shows the experimental results of this strategy on the Data_ D data set. In the experiment depicted in Figure 9, the registration set consists of four normal walking sequences from each sample, while the verification set consists of the latest two normal walking sequences.

The experimental recognition rate of Data_ *D* data set is shown in Figure 10. The experimental results in Figure 10 are used to evaluate the single angle of view.

The results show that the method proposed in this paper has obvious advantages for gait recognition with view changes. This means that the GAN model can generate better features and is robust to the change of viewing angle.

In order to better verify the performance of the model, several methods with better recognition effect (SVM, PSO, and PSO-SVM) were selected for comparison, and the experimental results are shown in Figure 11.

Compared with other methods, the model in this paper achieves better results from every angle, and the recognition rate is better than other methods. Under all test set angles, compared with the three methods in Figure 11, the best average recognition rate is obtained. The average recognition rates of the model in this paper are 93.24, 98.24, and 97.93 at 50°, 90°, and 120°, respectively, which shows that the model in this paper has good stability, can effectively deal with various test set angles, and maintains a high recognition rate.

## 5. Conclusions

Gait recognition, as a biometrics research center, has a wide range of applications in intelligent monitoring, human-computer interaction, security, and other fields, each with its own set of benefits. Computer vision technology can be used by experts in a variety of settings, such as competition refereeing, beginner dancer teaching, and dancer motion correction, to recognize motion in dance video images. In this research, we propose using GAN to dynamically recognize the gait contour of dancing motions. The average identification rates of this model at 50°, 90°, and 120°, respectively, are 93.24, 98.24, and 97.93, indicating that the recognition accuracy of the dance movement recognition approach is good. Simultaneously, a comparison of this strategy to other existing ways demonstrates that it is both successful and practicable. Although GAN is good at extracting contour data, dynamic features are crucial for gait identification. This paper suggests studying between frames, and I believe there is a bright future ahead.

## Figures and Tables

**Figure 1:** Change diagram of arch *x*, *y* displacement.

**Figure 2:** Synthesis of gait energy diagram.

**Figure 3:** Example figure of posture after returning to one.

**Figure 4:** Algorithm flow chart.

**Figure 5:** Divide the gait contour points of dancers based on.

**Figure 6:** Real-time action recognition process.

**Figure 7:** Walking state.

**Figure 8:** Comparison of the results of several recognition methods in the recognition of segmented actions.

**Figure 9:** The training set includes three walking conditions.

**Figure 10:** Recognition rate from four perspectives on Data_ D data set.

**Figure 11:** Recognition rate under different test set angles.

**Table 1:** Settings of encoder in generator.

Layers	Number of convolution kernels	Convolution kernel size	Step length	Batch processing	Activation function
Conv.1	98	5× 5× [1, 3]	4	N	L-ReLU
Conv.2	188	5 × 5 × 99	4	Y	L-ReLU
Conv.3	364	5 × 5 × 193	4	Y	L-ReLU
Conv.4	779	5 × 5 × 384	4	Y	L-ReLU

**Table 2:** Settings of decoder in generator.

Layers	Number of convolution kernels	Convolution kernel size	Step length	Batch processing	Activation function
F-Conv.1	779	5 × 5 × 384	1/4	Y	L-ReLU
F-Conv.2	364	5 × 5 × 193	1/4	Y	L-ReLU
F-Conv.3	188	5 × 5 × 99	1/4	Y	L-ReLU
F-Conv.4	98	5 × 5 × 3	1/4	N	Tanh

**Table 3:** Recognition result under two scheme.

Data set	Plan	Recognition accuracy
Data_ S	Method base on whole-body segmentation	0.869
	Methods of this paper	0.941
Data_ D	Method base on whole-body segmentation	0.712
	Methods of this paper	0.924

## Data Availability

The data used to support the findings of this study are available from the corresponding author upon request.
